The article "Clinical Evaluation of Efficacy on Ultrasound Combined with Neuromuscular Electrical Stimulation in Treating Lumbar Disc Herniation" was retracted in 2023. Reasons: signs of a paper mill; compromised peer review; unreliable results or conclusions.

# Clinical Evaluation of Efficacy on Ultrasound Combined with Neuromuscular Electrical Stimulation in Treating Lumbar Disc Herniation

**DOI:** 10.1155/2022/1822262

**Published:** 2022-09-26

**Authors:** Jingjing Chen, Binbin Han, Junqiu Du, Yudong Lu

**Affiliations:** ^1^Department of Rehabilitation Medicine, Lianshui County People's Hospital, Huai'an, Jiangsu 223400, China; ^2^Department of Rehabilitation Medicine, The Affiliated Huai'an Hospital of Xuzhou Medical University (Huai'an Second People's Hospital), Huai'an, Jiangsu 223002, China

## Abstract

**Purpose:**

To investigate the clinical efficacy of ultrasound (US) combined with neuromuscular electrical stimulation (NMES) in treating lumbar disc herniation (LDH) and its effect on the level of inflammatory factors.

**Methods:**

The data of 240 patients with LDH treated at our hospital from January 2020 to February 2021 were reviewed and classified into an US combined with NMES treatment group (US+NMES, *n* = 80), NMES only treatment group (NMES, *n* = 80), and US only treatment group (US, *n* = 80). Their Visual Analogue Scale (VAS) and Oswestry Disability Index (ODI) scores, levels of inflammatory factors and pain mediators, recovery rate, and total recovery time before and after treatment were compared. Additionally, the incidence of complications/adverse reactions was also investigated.

**Results:**

Compared with data before treatment, the three groups had lower VAS and ODI scores, inflammatory factor levels (interleukin- [IL-] 1, IL-6, and tumor necrosis factor- [TNF-] *α*), and pain mediators (transforming growth factor- [TGF-] *β*1, prostaglandin E2 [PEG2], and 5-hydroxytryptamine [5-HT]) after treatment, with the most significant decrease observed in the US+NMES group. Compared with patients who received US or NMES treatment alone, patients from the US+NMES had faster recovery time and lower incidence of complications/adverse reactions.

**Conclusion:**

Collectively, US combined with NMES was associated with significant relief in pain and lumbar dysfunction and reduced local inflammatory response and pain mediator levels in LDH patients, suggesting that this combined approach could achieve better efficacy than US or NMES alone.

## 1. Introduction

Lumbar disc herniation (LDH) is the most common disease in orthopedics, mostly induced by a sedentary lifestyle or strain [1]. It occurs in more than 60% of patients with low back and leg pain and is also one of the most frequent diseases undergoing spine surgery [2]. LDH can lead to lumbar and leg pain clinical symptoms, which affect lumbar activity. Additionally, it can be accompanied by unilateral/bilateral lower extremity pain and numbness or radiating pain in the lower extremities [3], seriously impacting the life and work of patients [4]. Current studies have shown that the pathogenesis of LDH is related to mechanical compression; that is, the nerve root is subjected to mechanical compression, causing the nucleus pulposus to protrude into the spinal canal and therefore causing acute compressions on nerve roots. The degree of herniation has been positively related to the degree of pain. In addition, its pathogenesis is also associated with inflammatory responses, whereby the protruded nucleus pulposus serves as a biochemical and immunological stimulus to produce inflammation in the surrounding tissues and nerve roots. As previously reported, the levels of serum inflammatory factors are increased in patients with LDH [5]. The immunoinflammatory mechanism is crucial for the occurrence and development of neuropathic pain. Inflammatory cell infiltration and immune cell activation can stimulate the generation and secretion of various inflammatory mediators, while the immune response of anti-inflammatory factors is more active in damaged nerves and dorsal root ganglions [6, 7]. Monoamine neurotransmitters are also involved in the biochemical stimulation of nerve roots in LDH [8]. Currently, the main treatment measures for LDH include surgical treatment and nonsurgical options such as bed rest, nonsteroidal anti-inflammatory drugs (NSAIDs), and physiotherapy. Most patients can be relieved or cured by nonsurgical treatment, while 10%-15% of patients require surgical treatment [9]. NSAIDs are the first-line drugs for pain management in LDH but are often associated with complications such as gastrointestinal adverse reactions and unsatisfactory analgesic effects. Further, many patients are reluctant to undergo surgical treatment due to extensive trauma, high risk of postoperative complications, high cost, and long recovery time. Therefore, there is still an urgent need to find new treatments for LDH.

The article "Clinical Evaluation of Efficacy on Ultrasound Combined with Neuromuscular Electrical Stimulation in Treating Lumbar Disc Herniation" was retracted in 2023. Reasons: signs of a paper mill; compromised peer review; unreliable results or conclusions.

Some studies have reported that ultrasound with mechanical wave, cavitation, diffusion, and thermal effects contribute to local blood and lymphatic circulation and the inhibition of nerve fiber adhesion, thus achieving nerve repair [10]. Ultrasound can also improve the pain threshold of peripheral nerves and has a significant analgesic effect on neuritis and neuralgia [10]. Neuromuscular electrical stimulation (NMES), as a physical therapy, involves using a low-frequency pulse current to stimulate nerves and muscles and generate muscle contraction by peripheral neuron depolarization at neuromuscular junctions (motor end plates). Such stimulation can improve local blood circulation and motor function and exert analgesic function [11]. Ultrasound combined with NMES therapy is a new physical therapy approach. It is widely used in the clinical treatment of LDH because of its advantages of being noninvasive, less pain, and having few side effects. However, studies comparing the significance of ultrasound+NMES with ultrasound or NMES alone are lacking.

This study is aimed at investigating the clinical efficacy of ultrasound+NMES and assessed its effects on serum inflammatory cytokine levels and pain mediators in LDH patients compared with ultrasound or NMES alone to provide a reference for the clinical treatment of LDH.

## 2. Materials and Methods

### 2.1. Patient Information

In this retrospective study, the data of 279 patients diagnosed with LDH at our hospital from January 2020 to February 2021 were retrieved and assessed. Informed consent was obtained from all patients, and this study was approved by the Ethics Committee of Lianshui County People's Hospital (LSYYLL-2021JS-028).

The inclusion criteria of this study were as follows: (1) aged 18-70 years old and with good compliance, (2) diagnosed with LDH based on clinical manifestations and lumbar spine computed tomography (CT) or magnetic resonance imaging (MRI) examinations, mainly presenting with regular lower back pain, and (3) nonacute patients: with a disease duration > 1 month and lower limb flexion in straight leg raise test < 70°. The exclusion criteria were as follows: (1) patients with spinal tumors, spinal tuberculosis, lumbar spine fractures, spinal stenosis, severe osteoporosis, lumbar spondylolisthesis, and other complex low back pain; (2) patients with severe heart, liver, and kidney dysfunction or lumbar space-occupying lesions; (3) patients with infectious or autoimmune system diseases, mental illness, and diseases differentiated from LDH such as third lumbar transverse process syndrome and piriformis muscle injury; and (4) pregnant or breastfeeding patients.

A total of 240 patients were included in the study according to the criteria and randomly divided into an ultrasound combined NMES treatment group (US+NMES, *n* = 80), NMES only treatment group (NMES, *n* = 80), and ultrasound only treatment group (US, *n* = 80).

### 2.2. Treatment Methods

Patients in the three groups were all given conventional treatment (i.e., massage, traction, and anti-inflammatory painkillers). Based on the conventional treatment, the US+NMES group was also given ultrasound combined with NMES, while the NMES group received NMES only, and the US group received ultrasound therapy only before treatment and the 1st, 3rd, and 6th months after treatment, 2 times/d.

All treatments were completed by professional therapists following the same standard procedure. NMES was performed using the Xiangyu Medical XY-K-STSS-A neuromuscular low-frequency electrical stimulator, targeting both sides of the spinous process corresponding to a diseased intervertebral disc. The stimulation frequency range was 20~50 Hz, and the stimulation sequence was held for 6 × 5 s each time, with 10 s intervals between stimuli. Ultrasound therapy was performed by positioning the probes at the points with maximum tenderness on both sides of the lumbar spine, and the most suitable intensity (800-1000 KHz) was selected according to the patient's tolerance. Treatment time was 8-10 minutes each time.

The article "Clinical Evaluation of Efficacy on Ultrasound Combined with Neuromuscular Electrical Stimulation in Treating Lumbar Disc Herniation" was retracted in 2023. Reasons: signs of a paper mill; compromised peer review; unreliable results or conclusions.

### 2.3. Scoring Criteria

The Visual Analog Scale (VAS) and the Oswestry Disability Index (ODI) were used before treatment and in the 1^st^, 3^rd^, and 6^th^ months since starting treatment. The former scale quantified patient pain level based on the following: a 10 cm line with “0” on the left end suggesting “no pain” and “10” on the right end representing “unbearable pain.” The ODI includes 10 items (such as pain intensity), with a full score of 50 points. Higher scores indicated higher levels of lumbar dysfunction [12].

### 2.4. Enzyme-Linked Immunosorbent Assay (ELISA)

In each group, 3 ml of cubital venous blood was drawn from the patients before treatment and on the 1st, 3rd month, and 6th month after treatment. The collected blood was placed in dry vacuum red blood collection tubes without additives. After keeping at room temperature for 2 hours, the blood was centrifuged at 4000 r/min for 10 min to extract the supernatant. Corresponding ELISA kits were used to detect the levels of inflammatory factors (interleukin- [IL-] 1, IL-6, and tumor necrosis factor- [TNF-] *α*) and pain mediators (transforming growth factor- [TGF-] *β*1, prostaglandin E2 [PEG2], and 5-hydroxytryptamine [5-HT]).

### 2.5. Treatment Recovery Time and Occurrence of Complications/Adverse Reactions

The number of patients who recovered in the 1st, 3rd, and 6th months after treatment and the overall recovery time was recorded. Additionally, the incidence of complications/adverse reactions of the patients during a 1-year follow-up was also recorded.

### 2.6. Statistical Analysis

SPSS 26.0 was used for data processing and statistical analysis. Quantitative data with normal distribution was expressed as mean ± standard deviation (SD), and one-way ANOVA with Dunnett's posttest or Tukey's correction was used for multiple comparisons. Categorical data was expressed as frequency (*n*) or rate (%), and the chi-square test was used for statistical analysis. *P* < 0.05 was regarded as a significant difference.

The article "Clinical Evaluation of Efficacy on Ultrasound Combined with Neuromuscular Electrical Stimulation in Treating Lumbar Disc Herniation" was retracted in 2023. Reasons: signs of a paper mill; compromised peer review; unreliable results or conclusions.

## 3. Results

### 3.1. General Information about Patients

In all, the data of 279 patients meeting the study criteria were retrieved. After excluding 12 due to refusal to participate, 19 due to abandonment midway, and 8 for other reasons, a total of 240 patients were included in this study. They comprised of 88 males and 152 females, with an average age of 48.50 ± 10.54 years. Before treatment, there was no statistically significant difference among the groups in age, gender, race/nationality, height, weight, education level, marital status, course of the disease, use of pain reliever, primary complications, medical history, and family history (*P* > 0.05), suggesting that the basic characteristics of the three groups were well balanced (Table 1).

### 3.2. Ultrasound Combined with NMES Significantly Reduces Pain and Lumbar Dysfunction in Patients

VAS and ODI scores were used to evaluate the effect of US combined with NMES on pain and lumbar dysfunction in patients. The results showed that the VAS and ODI scores of the three groups in the 1st, 3rd, and 6th months after treatment were significantly lower than those before treatment, with the most significant reduction observed in the US+NMES group (*P* < 0.05; Figure 1). These findings suggested that ultrasound combined with NMES therapy was more effective than ultrasound or NMES alone in reducing pain and lumbar dysfunction in LDH patients.

### 3.3. Ultrasound Combined with NMES Significantly Reduces the Levels of Serum Inflammatory Factors and Pain Mediators in Patients

The levels of inflammatory factors and pain mediators in the serum of the patients were detected. The results showed that the levels of inflammatory factors (IL-1, IL-6, TNF-*α*) and pain mediators (TGF-*β*1, PEG2, 5-HT) in the three groups were significantly lower than before treatment and demonstrated a time-dependent decrease (*P* < 0.05). The US+NMES group had the most significant marker level reduction (Figures 2(a)–2(f)). These findings suggested that all three treatment methods could reduce the levels of inflammatory factors and pain mediators, but ultrasound combined with NMES had the best effects.

### 3.4. Ultrasound Combined with NMES Significantly Reduces the Recovery Time of Patients

Here, the recovery of patients in the 1st, 3rd, and 6th months after treatment was assessed. No significant difference was found among the three groups in the number of patients recovered in the 1st month after treatment, while the number of recovered patients in the US+NMES group was significantly higher than that in the other two groups in the 3rd and 6th months after treatment. In addition, the patients in the US+NMES group had the shortest overall recovery time (60.31 ± 28.38 days) (Table 2).

The article "Clinical Evaluation of Efficacy on Ultrasound Combined with Neuromuscular Electrical Stimulation in Treating Lumbar Disc Herniation" was retracted in 2023. Reasons: signs of a paper mill; compromised peer review; unreliable results or conclusions.

### 3.5. Ultrasound Combined with NMES Significantly Reduces the Incidence of Complications/Adverse Reactions in Patients

After a one-year follow-up, the incidence of complications/adverse reactions, such as low back pain, sciatica, and intermittent claudication, in the three groups was investigated. Patients from the US+NMES group had the lowest incidence of complications/adverse reactions, followed by the US and NMES groups (Table 3). In addition, no cauda equina syndrome occurred in the combined group. Collectively, compared with the other two treatments, ultrasound combined with NMES demonstrated greater efficacy in reducing the incidence of complications/adverse reactions in LDH patients.

## 4. Discussion

Relevant clinical practice guidelines of the American College of Physicians and the United States Department of Defense [13, 14] indicate that conservative treatments such as NMES, ultrasound, transcutaneous electrical nerve stimulation, acupuncture, and massage can achieve the expected therapeutic effect in most patients with low back pain. Li et al. [15] summarized the literature on electrical stimulation for LDH published at home and abroad in the past decade and reported that electrical stimulation had a clear effect on LDH. Wu et al. [16] found that ultrasound and sling exercise therapy could effectively treat LDH in randomized clinical trials. Further, the combination of electrical stimulation and ultrasound was investigated and was found to be effective in the treatment of postherpetic neuralgia [10] and knee arthritis. Our study also found that the combined use of ultrasound and NMES, and even when the two treatments were used alone, could reduce the VAS and ODI scores of the patients, but the combination treatment had better efficacy.

TGF-*β*1 is also a differentiation and growth regulator with multiple functions and plays a vital role in inflammatory response and tissue repair [17]. 5-HT is a monoamine released by platelets and mast cells after tissue damage. It can directly stimulate sensory nerve fibers and interact with other inflammatory mediators to exert synergistic injurious effects through 5-HT2A receptors [18]. This study found that ultrasound combined with NMES could significantly reduce the serum levels of inflammatory factors IL-1, IL-6, and TNF-*α* and pain mediators TGF-*β*1, PEG2, and 5-HT levels, and the effects were superior than ultrasound or NMES alone. Therefore, these observations suggest that the combined therapy had more advantages in regulating inflammatory mediators. The underlying mechanism can be hypothesized to relate to the following three aspects. First, pulsed radiofrequency prevents pain signals from passing through nerves and continuously inhibits the induced synaptic activity, thereby producing pain inhibition [19]. Second, the field effect of the combination approach inactivates inflammatory mediators around damaged nerves, improves local blood circulation, and repairs damaged nerves [20]. Third, ultrasound and NMES can synergize and complement each other to enhance treatment efficacy.

The article "Clinical Evaluation of Efficacy on Ultrasound Combined with Neuromuscular Electrical Stimulation in Treating Lumbar Disc Herniation" was retracted in 2023. Reasons: signs of a paper mill; compromised peer review; unreliable results or conclusions.

The results of this study were consistent with a study by Yang et al. [20]. Studies have shown that LDH after degenerative abnormalities resulted in granulation tissues with inflammatory changes, which can produce many inflammatory factors and further aggravate degeneration [21]. Therefore, we speculate that the direct and effective suppression of pain mediators (TGF-*β*1, PEG2, 5-HT) levels by the combination treatment might be related to the inhibition of local degeneration and thus a reduction in their involvement in disease progression. In terms of recovery time and incidence of complications/adverse reactions, the combined treatment group was significantly better than the other two groups, suggesting that ultrasound combined with NMES could contribute to strengthening anti-inflammatory and analgesic effects and improving tissue repair and patients' prognoses.

Despite the interesting observations reported, there were some shortcomings worth describing. First, this study could have contained some unwilling and unavoidable bias due to its retrospective and single-center design. Second, although 240 cases were investigated, the number of cases allocated to each group might have been limited. Third, the treatment periods were quite long, and there could have been some unrecorded interfering factors, which could not be verified due to the retrospective nature of this study. Thus, larger cohort studies using prospective, randomized, and multicenter settings are required to further validate these findings.

## 5. Conclusion

In conclusion, ultrasound combined with NMES therapy was associated with a significant reduction in the local inflammatory response in LDH patients, improvements in functional impairment, low back pain and pain in the lower extremities, and had fewer complications/adverse reactions. However, further investigations using prospective and randomized settings are required to confirm our findings and provide concrete evidence for its potential clinical implementation because this approach is comparatively simple and noninvasive and has demonstrated promising efficacy.

## Figures and Tables

**Figure 1:** Effects of three treatment methods on pain and lumbar dysfunction in patients. (a. b) VAS scores and ODI scores before and after treatment. *N* = 80 per group. Data were expressed as mean ± SD. ^∗∗^*P* < 0.01 vs. NMES group, ##*P* < 0.01 vs. US group; US: ultrasound; NMES: neuromuscular electrical stimulation; VAS: Visual Analog Scale; ODI: Oswestry Disability Index.

The article "Clinical Evaluation of Efficacy on Ultrasound Combined with Neuromuscular Electrical Stimulation in Treating Lumbar Disc Herniation" was retracted in 2023. Reasons: signs of a paper mill; compromised peer review; unreliable results or conclusions.

**Figure 2:** Effects of three treatments on serum inflammatory factors and pain mediator levels in patients. (a)–(f) ELISA for detecting serum levels of IL-1 (a), IL-6 (b), TNF-*α* (c), TGF-*β*1 (d), PEG2 (e), and 5-HT (f); *N* = 80 per group. Data were expressed as mean ± SD. ^∗∗^*P* < 0.01 vs. 0 (month) in each group, ##*P* < 0.01; US: ultrasound; NMES: neuromuscular electrical stimulation.

**Table 1:** Baseline characteristics of the included patients (*n* = 240).

Variables	Treatment groups				
	US+NMES group (*n* = 80)	NMES group (*n* = 80)	US group (*n* = 80)	*t/χ* ^2^	*P*
Age (year) (mean ± SD)	49.15 ± 10.03	48.30 ± 9.22	48.04 ± 12.23	0.242	0.785
Gender (*n*)				0.467	0.792
Male	30	31	27		
Female	50	49	53		
Nationality (*n*)				0.173	0.917
Han ethnicity	65	66	67		
Minorities	15	14	13		
Height (mean ± SD)	166.90 ± 7.71	166.81 ± 6.53	167.25 ± 6.51	0.089	0.915
Weight (mean ± SD)	63.15 ± 14.04	63.04 ± 12.74	62.45 ± 12.77	0.0064	0.938
Education level (*n*)				4.605	0.595
Middle school	43	46	38		
High school	30	22	33		
College	4	7	6		
Master degree	3	5	3		
Marital status (*n*)				2.275	0.321
Married	13	14	20		
Single	67	66	60		
Course of disease (*n*)				4.440	0.617
Low back pain	6	5	5		
Beginning of nerve compression	42	31	35		
Severe nerve compression	23	34	28		
Atrophy of innervating nerves	9	10	12		
Use of pain relievers (*n*)				3.879	0.144
Yes	57	61	67		
No	23	16	13		
Medical history (*n*)				4.183	0.124
Yes	59	69	61		
No	21	11	19		
Family history (*n*)				2.312	0.315
Yes	57	64	64		
No	23	16	16		

Data was expressed as mean ± SD or *n*. US: ultrasound; NMES: neuromuscular electrical stimulation; US+NMES: ultrasound combined with NMES.

**Table 2:** Comparison of postoperative recovery of three groups of patients.

Variables	Time since start of treatment			Total recovery time (day)
	One month	Three months	Six months	
US+NMES group (*n* = 80)	21	59	77	60.31 ± 28.38
NMES group (*n* = 80)	10	41	60	72.15 ± 31.21
US group (*n* = 80)	16	46	66	72.26 ± 32.61
*T/χ* ^2^	4.815	9.059	14.251	2.510/2.472
*P*	0.090	0.011	0.001	0.013∗/0.015#

Data was expressed as mean ± SD or *n*. ^∗^*P* < 0.05, US+NMES group vs. NMES group; #*P* < 0.05, US+NMES group vs. US group. US: ultrasound; NMES: neuromuscular electrical stimulation; US+NMES: ultrasound combined with NMES.

**Table 3:** Comparison of complications between the three groups of patients.

Variables	Treatment groups		
	US+NMES group, *n* = 80 (%)	NMES group, *n* = 80 (%)	US group, *n* = 80 (%)
Low back pain	4 (5.00)	15 (18.75)	10 (12.50)
Sciatica	3 (3.75)	12 (15.00)	9 (11.25)
Numbness in lower limbs	1 (1.25)	9 (11.25)	8 (10.00)
Decline in lower limb muscle strength	1 (1.25)	7 (8.75)	6 (7.50)
Cauda equina syndrome	0 (0.00)	5 (6.25)	2 (2.50)
Intermittent claudication	4 (5.00)	15 (18.75)	10 (12.50)

Data was expressed as *n* (%). US: ultrasound; NMES: neuromuscular electrical stimulation; US+NMES: ultrasound combined with NMES.

The article "Clinical Evaluation of Efficacy on Ultrasound Combined with Neuromuscular Electrical Stimulation in Treating Lumbar Disc Herniation" was retracted in 2023. Reasons: signs of a paper mill; compromised peer review; unreliable results or conclusions.

## Data Availability

The datasets generated during and analyzed during the current study are available from the corresponding author on reasonable request.

## Abbreviations

NMES: Neuromuscular electrical stimulation
LDH: Lumbar disc herniation
ODI: Oswestry Disability Index
TGF: Transforming growth factor
5-HT: 5-Hydroxytryptamine.
